# Software Defect Prediction Based on Hybrid Swarm Intelligence and Deep Learning

**DOI:** 10.1155/2021/4997459

**Published:** 2021-12-28

**Authors:** Zhen Li, Tong Li, YuMei Wu, Liu Yang, Hong Miao, DongSheng Wang

**Affiliations:** ^1^School of Electronic and Information, Jiangsu University of Science and Technology, Zhenjiang 212100, China; ^2^Reliability and Systems Engineering Open Group, Jiangsu University of Science and Technology, Zhenjiang 212100, China; ^3^School of Reliability and Systems Engineering, Beihang University, BeiJing 100191, China; ^4^School of Economics and Management, Jiangsu University of Science and Technology, Zhenjiang 212100, China; ^5^School of Computer and Science, Jiangsu University of Science and Technology, Zhenjiang 212100, China

## Abstract

In order to improve software quality and testing efficiency, this paper implements the prediction of software defects based on deep learning. According to the respective advantages and disadvantages of the particle swarm algorithm and the wolf swarm algorithm, the two algorithms are mixed to realize the complementary advantages of the algorithms. At the same time, the hybrid algorithm is used in the search of model hyperparameter optimization, the loss function of the model is used as the fitness function, and the collaborative search ability of the swarm intelligence population is used to find the global optimal solution in multiple local solution spaces. Through the analysis of the experimental results of six data sets, compared with the traditional hyperparameter optimization method and a single swarm intelligence algorithm, the model using the hybrid algorithm has higher and better indicators. And, under the processing of the autoencoder, the performance of the model has been further improved.

## 1. Introduction

Software defects are the potential causes of errors, failures, and crashes of software systems [1]. In the industry with very strict requirements on software quality and reliability, if the potential defects in the software are not eliminated in time, it may cause serious economic losses to enterprises, and even threaten people's life safety.

Software defect prediction technology gives the software development team more than an opportunity to detect the software defect module by spending more energy on the modules of defective tendency and spending less energy on the modules of no defective tendency [2]. The software will be a better utilization of resources of the project and also can greatly reduce the test work of manpower and material resources consumption, saving the cost of test and improving research and development efficiency.

In recent years, many researchers have carried out various studies on software defect prediction technology and proposed software defect prediction models based on machine learning and statistics, such as logistic regression, classification tree, multilayer perceptron, radial basis function, and support vector machine [3]. In 2000, Denaro [4] used logistic regression to estimate software defects on 37 indicators of antenna configuration software and found that static software metrics and the number of software defects had a certain correlation. The multilayer perceptron (MLP) proposed by Pizzi et al. [5] in 2002 is an effective software defect research technique. Mahaweerawa et al. [6] used fuzzy clustering to predict software defects for the first time in 2002 and applied radial basis function (RBF) to predict software defects. Menzies et al. [7] built a Bayesian network defect prediction model on the Promise dataset in 2004 and used PD and PF as performance indicators of evaluation results. Jindal et al. [8] established a neural network prediction model in 2014 to study software defects, and subsequently, various optimization models for the neural network were proposed, such as PSO-BP and SA-BP.

However, model optimization is one of the most difficult challenges in the implementation of machine learning algorithms, including hyperparameter optimization, data preprocessing, and feature extraction. In terms of model optimization, Soares et al. [8] developed and proposed optimization based on Pyelogram Analysis and Composed Exhaustive Search to find solutions for combinatorial optimization problems with different levels of difficulty. In the optimization algorithm research in literature [9], two improvements were made to the Cuckoo search (CS) algorithm to empower its capability in controlling the diversity of its population and enhance the exploration of CS. Literature [10] studied how to teach optimization technique (OT) courses in systems engineering curricula at the undergraduate level and proposed an approach based on experiments. In literature [11], the convergence speed of the algorithm was improved by combining strengths of self-assembly and the particle swarm optimization. Literature [12] proposed a new application of the metaheuristic Slime Mould algorithm (SMA) in the optimization and adjustment of interval type-2 fuzzy controller.

The aim of hyperparameter optimization is to find a set of hyperparameters which can make machine learning algorithm have the best performance in verifying the realization of data set. In order to realize efficient automatic processing of model selection and hyperparameter optimization and to establish a suitable nonlinear relationship model between software static measurement and defect, a swarm intelligence optimization algorithm is proposed for dynamic optimization and hyperparameter optimization of deep neural network models.

In order to further improve the accuracy and accuracy of prediction model positioning, this paper uses functional defect samples for training and continues to use autocoding for feature extraction after data preprocessing to reduce the dimension of data samples, remove redundant features, and improve the efficiency of deep learning training.

## 2. Concept and Method

At present, based on the difference of research objects and research results, software defect prediction technology is mainly divided into static software defect prediction technology and dynamic software defect prediction technology. This article studies static software defect prediction technology, which is to construct software defect prediction through historical data and metrics. The model is used to judge the defect tendency of the software module.

### 2.1. Static Software Defect Prediction Technology

The static software defect prediction technology is to analyze the software module code, design the corresponding measurement element, and establish a suitable software defect prediction model based on the measurement element through the analysis of the software defect history data and then use the established software defect. The prediction model performs software defect prediction. The prediction results usually include two types: defects (usually recorded as 1) and nondefects (usually recorded as 0), as shown in Figure 1.

There is an obvious nonlinear relationship between software static measurement data and software defects, which does neither obey the known mathematical model nor is it a simple combination of basic nonlinear relationship functions. Therefore, the nonlinear model of software static measurement and defect must have the self-learning ability based on the existing static measurement and defect data set, in order to adaptively obtain the nonlinear model and its parameters that conform to the relationship between the software static measurement and defect.

### 2.2. Data Set for Training

The software measurement and defect data consist of two parts. One part is the static measurement information of each function of the software, and the other part is the defect label (0 or 1) of each function of the software.

Considering the existing data set limited in amount of metrics and records, this paper expanded the static metrics based on common principle and TestBed and meanwhile developed a web crawler tool to get software code to be measured and fault information from open source software website.

#### 2.2.1. Static Metrics of Software

We concluded the static metrics based on common principle and TestBed which is a tool widely used for static analysis on software. The whole metrics is listed in Table 1.

#### 2.2.2. Cutting Software into Function

Process-oriented languages have strict syntax and semantic specifications and must meet formal programming and coding requirements for function definitions and code writing. These grammatical and semantic specifications provide slicing standards for code function-level slicing and provide an effective way to improve the accuracy of software defect prediction based on code function-level slicing technology. This article is based on the Clang analyzer to perform lexical and grammatical analysis of the code and implement function-level slicing to improve the accuracy of defect data location. The slicing steps are as follows:

  S1 (file filtering settings): CPP cutting includes the extraction of various files, including .c files and .cpp files
  S2 (configure clang analyzer): use clang analyzer to analyze CPP, compile C\C++ language into LLVM intermediate expressions, so as to realize lexical and grammatical analysis
  S3 (main function analysis): use the get_and_write function; there are two parameters, one is the source code file name abs_file_name to be parsed and the folder name abs_dir_name to be output.
  S4 (extract function analysis): First create a parser, read in the file, get, and analyze the cursor node unit in the syntax parse tree, use kind (the kind element represents the components of a node, for example, is this a class, a function, or a variable name, etc.), spelling (the name of the extracted function body, it can also be a class body, etc.), location (the file start line and file end line of the function body), get_children (get all the nodes in the cursor).
  S5 (determine whether it is the required function body or class body): after the judgment is completed, call write_fun to write to the file.
  S6 (exception handling): unable to name the overloaded function—use special characters and English meaning to reset the function name to replace it.

#### 2.2.3. Measurement and Merge into Data for Training

The following takes the process-oriented C language software as an example to illustrate the process of data acquisition based on web crawlers, as shown in Figure 2.

The process shown in Figure 2 mainly includes three aspects. The first is to use code slicing technology for C language to establish function-level software measurement results. The second is to use web crawler technology to automatically capture and identify the code and defect data of open source software websites. The third is to generate C language software metrics and defect data through data matching of function names. Self-developed software tools are used in the data generation process, which have the characteristics of fast speed, correct matching, high data quality and function-level data granularity, which can provide high-quality and efficient software metrics and defect data for software defect prediction models.

### 2.3. Deep Learning

Deep learning is a learning method that uses data to train and learn the deep neural network to extract the characteristics of a nonlinear model by constructing a neural network of multiple levels. After obtaining the data set composed of the metric element and defect information, the data set must be processed, analysed, and learned. The learning potential of the deep neural network on the data characteristics can dig out the nonlinear relationship between the data and obtain the metric element and the defect. The mapping logic of software, thereby establishes a nonlinear model of software static measurement metadata and defect prediction data.

#### 2.3.1. Deep Neural Network

A deep neural network (DNN) is a feed-forward artificial neural network [13], also known as a multilayer perceptron. According to the position of the node in the network, it can be divided into input layer, hidden layer, and output layer. Compared with the shallow network, DNN has multiple hidden layers, and each layer can also have a larger number of neural units. The output of the current hidden layer will be used as the input of the previous hidden layer or output layer.  Figure 3 is a schematic diagram of the structure of a fully connected deep neural network.

Correspondence exists between all variables in DNN. Suppose there is a DNN with *N* + 1th layers, where the input layer is the 0th layer, the hidden layers are the 1st to *N* − 1th layers, and the output layer is the *N*th layer. Exist *n* ∈ (0, N], for any *n*th layer, there is the following correspondence:

(1) $$\begin{array}{c} {\text{net}}_{k}^{n}=\sum_{i=1}^{N^{n-1}}\omega_{ik}^{n}\cdot z_{k}^{n-1}+b_{k}^{l}, \end{array}$$

(2) $$\begin{array}{c} z_{k}^{n}=f_{l}\left({\text{net}}_{k}^{n}\right), \end{array}$$

where net_*k*_^*n*^ is the input value of the *k*th node in the *n*th layer, *N*^*n*^ is the number of nodes in the *n*th layer, *w*_*ik*_^*n*^ is the weight between the *i*th node in the *n*th layer and the *k*th node in the nth layer, *z*_*n*_^*k*^ is the *n*th output value of the *k*th node in the layer, and *b*_*k*_^*l*^ is the bias of the *k*th node in the *n*th layer, and *f*_*l*_(·) is the activation function of the nth layer. For the activation function *f*_*l*_(·), different forms can be selected in different algorithms. Common activation functions include sigmoid function, softplus function, and rectified linear unit (ReLU) function.

Loss function, also known as objective function or error function, is mainly used to measure the error between the actual output of the network and the expected output, so as to guide the learning of network parameters. For regression problems, functions such as square loss are generally used; for classification problems, functions such as logarithmic loss and cross entropy are generally used. Different loss functions will affect the training speed and generalization ability of the network. In a binary classification problem like this paper, cross entropy is generally used as the loss function, and softmax is used as the activation function in the output layer of the model. Cross entropy is a very important concept in information theory, mainly used to measure the difference between two probability distributions. For the sample (*x*, *y*), *x* is the sample and *y* is the corresponding label, assuming that the set of values is {0, 1}. When the true label of a sample is *y*, and the probability of the sample label *y* = 1 is *p*, then the cross-entropy loss function of the sample is

(3) $$\begin{array}{c} \text{loss}=-\left(y\;\log\left(p\right)+\left(1-y\right)\log\left(p\right)\right). \end{array}$$

In order to minimize the error value of the loss function, backpropagation technology is used in the network to trace back from the output layer to the input layer and update the weights and biases according to the influence of different parameters. The commonly used method is the gradient descent algorithm, but there will be problems such as slow convergence, large fluctuations in the decline process of the loss function value, and falling into a local minimum.

This paper used the gradient descent optimization algorithm Adam, which is a method to calculate the adaptive learning rate for each parameter. It not only stores the exponential decay mean value of the past gradient square, that is *v*_*t*_ but also stores the exponential decay mean value of the past gradient, that is, *m*_*t*_. In this way, the sliding average of the gradient and the square of the gradient can make each update related to the historical value. The formula is as follows:

(4) $$\begin{array}{c} m_{t}=\beta_{1}m_{t-1}+\left(1-\beta_{1}\right)g_{t}, \end{array}$$

(5) $$\begin{array}{c} v_{t}=\beta_{2}v_{t-1}+\left(1-\beta_{2}\right)g_{t}^{2}, \end{array}$$

Adam's update rules are as follows:

(6) $$\begin{array}{c} \theta_{t+1}=\theta_{t}-\frac{\eta }{\sqrt{{\hat{v}}_{t}}+\in }{\hat{m}}_{t}. \end{array}$$

In formulas (4)∼(6), *η* = 0.001, *β*_1_ = 0.9, *β*_2_ = 0.999, and ∈ = 1*e* − 8 is to prevent the divisor from being 0, *g*_*t*_ represents the gradient, and the formulas of ${\hat{m}}_{t}$ and ${\hat{v}}_{t}$ are as follows:

(7) $$\begin{array}{c} {\hat{m}}_{t}=\frac{{\hat{m}}_{t}}{1-\beta_{1}^{t}}, \end{array}$$

(8) $$\begin{array}{c} {\hat{v}}_{t}=\frac{v_{t}}{1-\beta_{2}^{t}}. \end{array}$$

#### 2.3.2. Self-Encoding Network

Autoencoder (AE) is an unsupervised learning algorithm. The label is directly replaced by the input. Its learning method is shown in Figure 4.

The autoencoder can be considered as a neural network with only one hidden layer, which realizes the reconstruction of features through compression and restoration. The input data is a feature, the input layer to the hidden layer is an encoder, which can compress the input into a latent space representation; the hidden layer to the output layer is a decoder, which reconstructs the input from the latent space representation. The number of input and output neurons of the autoencoder is equal to the feature dimension. Train this autoencoder to make the output features and input features as consistent as possible. The autoencoder tries to reproduce its original input. Therefore, during training, the output in the network should be the same as the input, that is, *y* = *x*. Therefore, the input and output of an autoencoder should have the same structure. We use the training data to train this network. After the training is over, the network has learned the ability of *x* ⟶ *h* ⟶ *x*. For us, *h* at this time is very important because it is another expression of the original data without losing the amount of information as much as possible. Its structure is shown in Figure 5.

By training the autoencoder whose output value is equal to the input value, the potential representation *h* will have value attributes. One way to obtain useful features from a self-encoder is to limit the dimension of *h* to be smaller than the input *x*. In this case, it is called a loss self-encoder. By training the loss representation, the autoencoder can learn the most important features in the data.

### 2.4. Model Evaluation Indicators

In the research of typical defect prediction technology [14], the evaluation performance related to confusion matrix is usually used to evaluate the prediction results, such as accuracy, precision, recall, and F-measure (F-measure). The confusion matrix includes two columns, as shown in Table 2.

TP is the number of modules that are predicted to contain defects and are actually defective, FP is the number of modules that are predicted to contain defects and are actually free of defects, FN is the number of modules that are predicted to contain no defects and are actually defective, and TN is the number of modules that are predicted to contain no defects and are actually the number of modules without defects. Based on these four categories, the following concepts are introduced to evaluate the performance of the classifier.

(1) Accuracy: calculate the ratio of all correctly classified test cases (TP + TN) to the total number of test cases, namely,
  (9) $$\begin{array}{c} \text{accuracy}=\frac{\text{TP}+\text{TN}}{\text{TP}+\text{FP}+\text{FN}+\text{TN}}. \end{array}$$
Accuracy gives the overall effect of prediction and is one of the most commonly used indicators when evaluating classifier models. However, in the defect prediction, due to the serious class imbalance problem in the defect data, in fact, it is meaningless to use the accuracy as the evaluation index of the prediction model. Suppose there are 100 modules in a software project, of which 1 is a defective module and the remaining 99 are nondefective modules; at this time, if all software modules are predicted as nondefective modules, the accuracy of the prediction model will be as high as 99%, but in fact, the predictive model did not find the defective module. Therefore, in the current defect prediction, accuracy is no longer used as the evaluation index of the prediction model [15].
(2) Precision: calculate the ratio of the number of test cases (TP) correctly classified as positive to the number of all test cases classified as positive, namely,
  (10) $$\begin{array}{c} \text{precision}=\frac{\text{TP}}{\text{TP}+\text{FP}}. \end{array}$$
(3) Recall rate: calculate the ratio of the number of test cases (TP) correctly classified as positive to the actual number of positive test cases, namely,
  (11) $$\begin{array}{c} \text{recall}=\frac{\text{TP}}{\text{TP}+\text{FN}}. \end{array}$$
(4) F-measure: it can be seen from the definition that a pair of opposite evaluation indexes of recall rate and precision rate. But a good software defect prediction model should have a high recall rate and precision rate at the same time. Therefore, when evaluating the effect of the software defect prediction model, it is necessary to combine the recall rate with the precision rate. This is the F-measure evaluation index, and the calculation formula is
  (12) $$\begin{array}{c} \text{F}-\text{measure}=\frac{\left(\left(1+\beta^{2}\right)*\text{recall}*\text{precision}\right)}{\beta^{2}*\text{recall}*\text{precision}}, \end{array}$$
where*β* represents the importance of recall and precision, usually take 1, which means that the two are equally important, denoted as F1.
(5) AUC (area under the ROC curve): in the two-class model, the AUC indicator is often used as the most important evaluation indicator to measure the accuracy of the model in the model evaluation stage. AUC considers the ranking quality of model predictions, reflecting the ratio of positive examples ahead of negative examples by the model.

## 3. Hyperparameter Optimization Based on Hybrid Wolf Pack Algorithm

In the deep learning model, the most important thing is “parameter tuning.” Some parameters, such as weights and biases, will be optimized as the model is trained, and some parameters cannot be optimized during model training. These are hyperparameters. They often determine the framework and settings of the model, so optimization should be started before the model is trained. The choice of hyperparameters can directly affect the performance of the algorithm model, but the hyperparameter optimization process often depends on the accumulation of professional knowledge and long-term experience. Therefore, research to find suitable hyperparameter optimization methods is an important factor that affects the effect and efficiency of deep learning algorithms [16].

At present, hyperparameter optimization methods are mainly divided into grid search, random search, and other directional searches. Grid search is to adjust the parameters according to the step length within the specified parameter range and train the learner based on the adjusted parameter set, so as to find the parameter set that can maximize the model accuracy among all the parameters. Random search is not trying all possible combinations, but random combinations. This method is similar in nature to grid search, except that the change in the gap between parameters is random and not necessarily equal. It is a random selection of values for each hyperparameter. In all candidate parameter sets, through loop traversal, try every possibility, and the best performing parameter set is the final result.

Grid search requires traversal of all possible parameter combinations within the parameter range, which is also its disadvantage. When there are more data sets and multiparameters, this approach will cause the number of calculations to increase exponentially, which will consume a lot of time, and ultimately there is no guarantee that perfect hyperparameter values can be found. Although random search has a relatively higher chance of finding the optimal parameters than grid search, when the parameter dimension becomes larger, it is the same as the grid search, and the amount of calculation that surges is also time-consuming. In short, these two search methods are only permutation and combination of parameters, which belong to violent exhaustive search methods, so they will inevitably sacrifice a lot of time and computing power, and they cannot point out the optimization direction for subsequent better parameter searches.

Hyperparameter optimization is a dynamic process, but grid and random search can only combine different parameters and cannot dynamically select and adjust parameters according to the training state of the model and allow the parameters to actively approach the optimal value. Therefore, some researchers have proposed the use of swarm intelligence algorithms for hyperparameter optimization. Zhang optimized the hyperparameters based on the group directional optimization method of improved particle swarm algorithm. It is mainly through the mutual cooperation and information sharing of particle swarms to determine the update of hyperparameters. Therefore, this search method based on swarm intelligence algorithm can avoid grid and random blindness problems and can ensure that the parameters are gradually optimized as the algorithm runs [17]. Similarly, the use of improved particle swarm algorithm for hyperparameter optimization is also studied in [18]. The improvement idea is to adjust the algorithm in time when it is found that the algorithm may be in a stagnant state, thereby speeding up the algorithm's convergence speed. At the same time, because the hyperparameter optimization problem is a nonlinear problem, there will be many local optimal solutions. Li avoids the algorithm from falling into the local optimal solution by adding disturbance to the global optimal. However, this improvement does not greatly increase the accuracy of the algorithm because the update strategy of the particle swarm algorithm is too simple, and it is difficult to ensure the optimization ability of the particles using only this update method. Therefore, when the algorithm is improved, it can be integrated into the search methods of other suitable agents. The search category of agents is increased through algorithm mixing, and different local solution spaces are searched based on multiple agents, so as to solve the problem that hyperparameter optimization is easy to fall into local optimal solutions.

In order to achieve fast and accurate hyperparameter optimization, this paper studies the optimization of the hyperparameters of the deep neural network model based on the hybrid swarm intelligence algorithm. First, according to the characteristics of the particle swarm algorithm and the Wolf Pack algorithm, the two are mixed to obtain an improved hybrid Wolf Pack algorithm. Then when using the swarm intelligence algorithm to optimize the hyperparameters, the loss function of the model is used as the standard for supervising the state of the model, and the value of the loss function is taken as the value of the fitness function in the swarm intelligence algorithm. Through the iterative search of the agent, an optimal set of hyperparameters is found, thereby improving the software defect prediction performance of the deep neural network model.

### 3.1. Swarm Intelligence Algorithm

#### 3.1.1. Particle Swarm Algorithm

Particle swarm optimization (PSO) realizes the search for the optimal solution based on the mutual cooperation and information sharing among particles in the swarm. First, the initial population is randomly generated, and the fitness value of each particle is determined by the objective function. The fitness value represents the quality of the particle position. In each iteration of the search for the optimal solution, each particle will adjust its position following two extreme values. One is the optimal fitness value found so far by the particle itself, which is called the individual extreme value. The other is the optimal fitness value found so far by all other particles in the population, which is called the global extremum.

The mathematical expression of the particle swarm optimization algorithm is as follows: in a dimensional search space, there is a population of *m* particles, that is, *X* = {*X*1,…, *X*_*i*,…, *X*_*m*}, the position of the *i*th particle is expressed as *X*_*i* = {*X*_*i*1, *X*_*i*2,…, *X*_id}^*T*^ and its speed is expressed as *V*_*i* = {*V*_*i*1, *V*_*i*2,…, *V*_id}^*T*^. The individual extremum of the *i*th particle is expressed as *P*_bi = {*P*_bi1, *P*_bi2,…*P*_bid}^*T*^, and the global extremum of the population is expressed as *g*_b = {*g*_b1, *g*_b2,…, *g*_bd}^T^. The particles update their velocity and position according to formulas (13) and (14):

(13) $$\begin{array}{c} v_{id}^{\left(t+1\right)}=wv_{id}^{t}+c_{1}{\text{rand}}_{1}\left(\;\right)\left(P_{bid}^{t}-x_{id}^{t}\right)+\;c_{2}{\text{rand}}_{2}\left(\;\right)\left(g_{bd}^{t}-x_{id}^{t}\right), \end{array}$$

(14) $$\begin{array}{c} x_{id}^{\left(t+1\right)}=x_{id}^{t}+v_{id}^{\left(t+1\right)}. \end{array}$$

In the formula, *w* is the inertia weight, which is a nonnegative number in [0, 1], which represents the ability of the particle to inherit the current speed; the learning factor c_1 and c_2, generally, represents the ability of the particle to learn; rand_1 ()and rand_2 () are random numbers belonging to (0,1). The update speed of the particle is composed of three parts. The first part is the previous speed of the particle, which represents that the current state of the particle is inertially moved by its own speed, which balances global exploration and local development capabilities; the second part is the “cognition” part, which represents the optimal position that the particle has experienced so far, and the difference between it and the current position of the particle represents the influence value of the particle's own experience on its next behavior; the third part is the “social” part, *g*_bd is the optimal position all particles so far found; the mutual cooperation and information sharing between the particles make the particles search in a better direction.

#### 3.1.2. Wolf Pack Algorithm

The Wolf Pack Algorithm (WPA) is intended to simulate the wolves' hunting behavior processing function optimization problem and divide the wolves into three categories: head wolves, detective wolves, and fierce wolves. The entire hunting activity of the Wolf Pack is abstracted into three intelligent behaviors (walking behavior, summoning behavior, and siege behavior), as well as the “victor is king” wolf generation rules and the “strong survival” Wolf Pack update mechanism.

(1) Criteria for the generation of wolves: start from a certain initial prey group in the space to be optimized, and the wolf with the best fitness value is used as the wolves.
(2) Wandering behavior: select the best *S*_num artificial wolves except the head wolves as the wolf detection to perform the wandering behavior. *S*_num is an integer selected randomly in [*n*(*α* + 1), *n*/*α*], *n* is the total number of artificial wolves in the Wolf Pack, and *α* is the wolf detection scale factor. First calculate the prey scent concentration at the current position of the detective wolf *i*. if *Y*_*i*_ < *Y*_lead_, then *Y*_lead_ = *Y*_*i*_. Detect Wolf replaces the position of the head wolf and initiate a summoning behavior; if *Y*_*i*_ > *Y*_lead_, detective wolf moves forward in *h* directions respectively (the step length at this time is called stepa). The position of the wolf *i* in the d-dimensional space after advancing along the *p*-th direction *p* = 1, 2, 3,…, *h*) is
  (15) $$\begin{array}{c} x_{id}^{p}=x_{id}+\sin\left(\frac{2\pi \times p}{h}\right)\times {\text{step}}_{p}^{d}. \end{array}$$
The detective wolf *i* keeps walking until the odor concentration perceived by a certain wolf *Y*_*i*_ < *Y*_lead_, or the number of walking *T* reaches the maximum *T*_max_.
Among them, there are differences in the prey search method for each wolf detection, that is, the value of is different, and it is the random integer taken in in [*h*_min_, *h*_max_] in the actual situation.
(3) Summoning behavior: the head wolf initiates a howling to perform the summoning behavior, and informs the surrounding fierce wolves to approach the head wolf quickly, where *M*_num = *n* − *S*_num − 1; when the fierce wolves hear howling, they all run quickly with a relatively long stride length. The ground is approaching the position of the head wolf (the step length at this time is called the raiding step length step_b_). Then, when the wolf *j* goes through the *k* + 1th iteration, the position in the d-dimensional space is
  (16) $$\begin{array}{c} x_{jd}^{k+1}=x_{jd}^{k}+{\text{step}}_{b}^{d}\cdot \frac{g_{d}^{k}-x_{jd}^{k}}{\left|g_{d}^{k}-x_{jd}^{k}\right|}, \end{array}$$
where *g*_*d*_^*k*^ is the position of the wolf of the *k*-th generation group in the d-dimensional space.
In the process of running, if the scent concentration *Y*_*j*_ < *Y*_lead_ perceived by the wolf *j*, then *Y*_*j*_ = *Y*_lead_ and the wolf *j* transforms into a head wolf and initiates a summoning behavior; if *Y*_*i*_ > *Y*_lead_, then the wolf *j* continues to carry out the raiding behavior, and when the distance between the wolf *j* and the head wolf *s*. *d*_is_ is less than the judging distance *d*_near_, it will be turned into a siege behavior. The judgment distance *d*_near_ is obtained by estimation:
  (17) $$\begin{array}{c} d_{\text{near}}=\frac{1}{D\cdot \omega }\cdot \sum_{d=1}^{D}\left|\max_{d}-\min_{d}\right|. \end{array}$$
Among them, *D* is the dimension of the variable space to be optimized; max_*d*_ and min_*d*_ are the maximum and minimum values of the *d*-th dimension space to be optimized. *ω* is the distance determination factor, and its different values will affect the convergence speed of the algorithm. When increases, it will accelerate the convergence of the algorithm, but if it is too large, it will make it difficult for artificial wolves to enter the siege behavior and lack the precision of prey search for.
(4) Siege behavior: the wolves conduct siege behavior according to formula (18). For the *k*-th generation of Wolf Pack, suppose the position of the prey in the *i*-th dimension space is *G*_*d*_^*k*^, and the following formula can be used to express the siege behavior of the Wolf Pack:
  (18) $$\begin{array}{c} x_{id}^{k+1}+\lambda \cdot {\text{step}}_{c}^{d}\cdot \left|G_{d}^{k}-x_{id}^{k}\right|, \end{array}$$
*λ* is the random number distributed in [−1, 1]; step_*c*_^*d*^ is the attack step length of artificial wolf *i* when it takes a siege behavior in the *d*-dimensional space.
The three types of intelligent behaviors include walking step length step_*a*_^*d*^, running step length step_*b*_^*d*^, attack step length step_*c*_^*d*^, and step length in the *d*-dimensional space involves the following relation:
  (19) $$\begin{array}{c} {\text{step}}_{a}^{d}=\frac{{\text{step}}_{b}^{d}}{2}=2\cdot {\text{step}}_{c}^{d}=\frac{\left|\max_{d}-{\text{main}}_{d}\right|}{S}. \end{array}$$
In the formula, *S* is the step length factor.
(5) The Wolf Pack update mechanism of “survival of the strong.” Eliminate the *R* artificial wolves with the worst objective function value, and generate *R* new artificial wolves randomly at the same time. The value of *R* is a random integer between [*n*/(2 × *β*), *n*/*β*] and *β* is the population update scale factor.

### 3.2. Hyperparameter Optimization Based on Hybrid Wolf Pack

#### 3.2.1. Hyperparameter

Hyperparameter optimization is also called hyperparameter adjustment. The deep learning algorithm contains thousands of parameters. Some of these parameters can be optimized by training, such as the weight in the neural network, which we call parameters. There are also some parameters that cannot be trained. To optimize, such as learning rate, we call it a hyperparameter (hyperparameter).

When training a neural network, it is essential to adjust the hyperparameters. This process can train a more efficient machine learning model more scientifically. The main optimized hyperparameters in this paper are the number of layers of the network, the number of neurons in each layer, and the learning rate.

- Number of network layers: in deep neural networks, in addition to the input layer and output layer, the number of hidden layers can be increased or decreased according to the learning situation. Adding a hidden layer can reduce network errors and improve accuracy, but it also complicates the network, thereby increasing the training time of the network and the tendency of “overfitting.”
- Number of neurons: after the training set is determined, the number of nodes in the input layer and the number of nodes in the output layer are determined accordingly. However, how to optimize the number of nodes in the hidden layer is a more difficult problem. Experiments show that if the number of hidden layer nodes is too small, the network will not have the necessary learning capabilities and information processing capabilities. On the contrary, if it is too much, it will not only greatly increase the complexity of the network structure and slow down the learning speed of the network but also the network is more likely to fall into a local minimum during the learning process.
- Learning rate refers to the magnitude of the update of the network weight in the optimization algorithm. The learning rate can be constant, gradually decreasing, momentum-based or adaptive. Different optimization algorithms determine different learning rates. When the learning rate is too large, the model may not converge, and the loss will continue to oscillate up and down; when the learning rate is too small, the model will converge slowly, and it will take longer to train.

#### 3.2.2. Hybrid Wolf Pack Algorithm

The PSO algorithm has a simple structure and few parameters and is easy to implement. Although the convergence speed is very fast at the initial stage of the iteration, it is easy to fall into the local optimization at the later stage of the iteration, leading to premature convergence. WPA has strong global exploration capabilities, especially in the later iterations, and will not fall into local optimum. Compared with PSO, WPA has lower randomness in the algorithm operation process, and the solution after running multiple times can be closer to the actual value and will not cause the solution value to deviate from the actual value in a large area. Based on the advantages and disadvantages of WPA and PSO algorithms, combining the two algorithms can achieve a good complementary effect [19]. The approach taken in the solution space is as follows: after the PSO algorithm particle search for particles, then use the wolf in the Wolf Pack algorithm. The search process of the group is refined again to determine the final new position.

The detailed process steps of the learning algorithm are as follows:

  S1: first initialize the parameters of the Wolf Pack algorithm and the particle swarm algorithm, calculate the fitness function, and update the individual extremum and the population extremum.
  S2: judge whether the current number of iterations meets the requirements, and if the number of iterations is not less than the minimum value, run down.
  S3: for each particle in the population, update the population according to the update formula of the particle swarm for their speed and position.
  S4: the wolf hunter wanders in directions, updates the position according to the wandering formula, and obtains the fitness value at the updated position.
  S5: find the updated optimal fitness value and optimal position of the head wolf.
  S6: the wolf initiates a summoning behavior, and the wolf runs towards the wolf according to the running formula.
(vii) S7: calculates the fitness value of the updated wolf, and updates the fitness value and position of the wolf at the current position.
  S8: given the number of raids, when the maximum number of raids is reached, the wolf becomes the head wolf, or *d*_is_ < *d*_near_. One of the three conditions is met, step 9 is executed, otherwise, step 6 is executed.
  S9: calculate and update the position of the siege wolf according to the formula, calculate the fitness value, and update the value of the current position.
  S10: according to the update mechanism of the Wolf Pack, execute the survival of the strong and discard the worst *R* wolf.
  S11: generate randomly wolves, and calculate the fitness value of wolves.
  S12: if the number of iterations does not reach the maximum requirement, turn to S2 to continue.

The maximum number of raids is set in S6 because when the positions of the wolf and the head wolf are difficult to meet *d*_is_ < *d*_near_, the running time of the algorithm becomes longer, and in severe cases, it may even fall into an infinite loop. Therefore, in order to shorten the running time of the algorithm, this paper determines the number of runs as 5 according to the value of the hyperparameter, the distance determination factor and the run step length, which can not only ensure that the wolf reaches the parameter search near the head wolf but also control the running time of the algorithm.

#### 3.2.3. Hybrid Wolf Pack Algorithm to Optimize Hyperparameters

In the hyperparameter optimization method, the manual tuning method requires a lot of experience and is relatively time-consuming; one disadvantage of grid optimization is that when multiple hyperparameters are involved, the number of calculations increases exponentially, and this method does not guarantee that the search will find the perfect hyperparameter value; the random optimization method has a relatively higher chance of finding the optimal parameter, but this method is suitable for low-dimensional data. In view of this situation, this article will use the hybrid Wolf Pack algorithm to optimize the hyperparameters. The flowchart is shown in Figure 6:

When the swarm intelligence algorithm is initialized, the dimensionality of the population in the hybrid algorithm is determined mainly by the number of hyperparameters that need to be optimized, and then the particle length is determined by the value range of each parameter. This paper takes the loss function of the deep neural network as the fitness function of the hybrid algorithm. Adjust and optimize the position of the particle, that is, the value of the hyperparameter, through the optimization of the fitness value. The purpose of this design is mainly to give full play to the powerful global optimization ability of the hybrid algorithm, so as to minimize the value of the loss function output by the deep neural network.

In the deep neural network in this article, we judge the current training state of the model by observing the monitoring indicators such as the value of the loss function during the training process and use the hybrid swarm intelligence algorithm to adjust the hyperparameters, so that the model can be used in a more scientific way. Effectively learn and train to improve the accuracy of model prediction.

## 4. Experimental Results and Comparison

In the current research, the establishment of a predictive model is mainly based on the measurement metadata with identified defect information, but in the actual process, the identified software measurement metadata is very poor [20]. At the same time, most of the current work results use public data sets, such as NASA's data sets. However, the limitation of the data sample size will have the problems of limited measurement elements, limited data amount, and relatively fixed sample set and training set, which makes the training effect poor. And, due to the simplification of the data set, the correctness, validity, and versatility of its defect prediction and location results cannot be guaranteed. Not only this, the quality and reliability of NASA's data sets have also been questioned by researchers. It is worth mentioning that the software warehouse on the Internet stores a large amount of software development and evolution data. In addition to source code and change logs, there are defect reports, etc., which can provide a large amount of sample data for software engineering prediction problems.

Different from the previous research using public data sets such as NASA, the data set used in this article is extracted through automated tools, crawling software defect information from open source websites and collating with the metric metainformation of the corresponding function. The experimental data sets in this article are all from C language software projects, in which the number of metric elements, that is, the number of features is 47, and the defect distribution is shown in Table 3.

### 4.1. Software Defect Prediction Model Based on Deep Neural Network

The premise of using a deep neural network to build a deep learning model is to determine the network settings such as the number of layers, the number of nodes, and the activation function of the network. In order to establish a software defect prediction model based on the deep neural network, this article will build the model and learn and train based on the Tensorflow framework. The flow chart is shown in Figure 7:

### 4.2. Feature Extraction Based on Autoencoder

The autoencoder learns the internal features of the data set by supervising itself, extracts useful feature information, and achieves the purpose of dimensionality reduction. This article will feed the data to the autoencoder before the deep neural network training. After the autoencoder training is over, the autoencoder obtains an effective data representation. At this time, the decoder is removed, and only the encoder is retained. Then, the output of the encoder will be directly used as the input of the subsequent software defect prediction model to complete the data dimensionality reduction, and the purpose of improving the training effect is achieved through this operation. The flow chart is shown in Figure 8:

### 4.3. Comparison of Different Hyperparameter Optimization Methods

The article realizes five optimization methods of hyperparameters—grid, random, particle swarm algorithm, Wolf Pack algorithm, and mixed Wolf Pack algorithm—and compares the 4 indicators of the model. The limits of the three hyperparameters solved in the experiment are as follows: the range of the number of hidden layers [2,6], the range of the number of nodes of the hidden layer [20,60], and the range of learning rate [1*e* − 4,1*e* − 2]; the rest parameter settings are as follows:

1. Grid optimization: set 45 parameter combinations within the range of hyperparameters. For example, the number of hidden layers is [2,3,4,5,6] and the number of nodes in the hidden layer is [25,40,55], the learn rate is [1*e* − 4,1*e* − 3,1*e* − 2].
2. Random optimization: the number of given parameter combinations in the hyperparameter range is 45.
3. Particle swarm optimization: the number of particles is 15, the maximum number of iterations is 3, learning factor *c*_1_=*c*_1_=0.5, and inertia weight *w*=0.9.
4. Optimization of Wolf Pack algorithm: the number of wolves is 15, the maximum number of iterations is 3, the distance determination factor is 8, the maximum number of travel restrictions is 3, the wolf detection scale factor *α*=3, the Wolf Pack update scale factor *β*=5, step factor *S*=20.
5. Hybrid Wolf Pack algorithm optimization: the parameters are the same as the particle swarm and Wolf Pack algorithms.

In the parameter setting of the above algorithm, the range of the three hyperparameters can be selected by the user. Each parameter setting of the grid optimization can be set randomly, but it is necessary to ensure that the final combination number is consistent with the random optimization and is equal to the product of the number of particles and the number of iterations of the particle swarm algorithm and the wolf swarm algorithm. For example, there are 45 (5 ∗ 3 ∗ 3) combinations in the above grid optimization, the number of parameter combinations for random optimization is set to 45, the number of particles in the particle swarm and wolf swarm algorithm is 15, and the number of iterations is 3. This is to ensure that the calculation amount of different algorithms is consistent, so as to ensure the credibility of the algorithm comparison results.

First, the data set is preprocessed, and the data is standardized and scaled. Next, each data set is divided into three parts, as the test set, training set and verification set, and then the software defect prediction model is trained using the training set and the verification set, and finally, the defect prediction is performed on the test set based on the trained model. Each group of experiments is trained 20 times, and the results are the average of 10 experiments. The experimental results are shown in Tables 4–9 and Figures 9–14.

The precision rate reflects the model's ability to distinguish negative samples, the recall rate reflects the model's ability to recognize positive samples, and the F-measure is a combination of the two. The larger the F-measure value, the more robust the classification model. AUC is the area under the ROC curve. The larger the value, the better the model.

Observing Tables 4–9 and Figures 9–14, it is found that compared with other methods, the optimization method of the hybrid algorithm (WPA-PSO) can not only ensure a higher precision rate but also improve the recall rate. As the overall evaluation index of the model, F-measure and AUC are also increasing with the improvement of optimization methods. In general, the superiority and inferiority ranking of hyperparameter optimization methods is WPA − PSO > WPA > PSO > random > grid.

### 4.4. Comparison of before and after Feature Extraction

The number of features of the dataset used in Section 4.1 is 47. These high-dimensional data will increase the complexity and reduce the accuracy of the model during data processing and construction of the training model. The article uses a self-encoding network with only one hidden layer and sets the number of nodes in the hidden layer to 32. The self-encoding network is trained through the training set, and finally the data set is re-encoded based on the trained self-encoding network. The encoded data set will continue to use five hyperparameter optimization methods to train the model. Each group of experiments is trained 20 times, and the results are the average of 10 experiments. The experimental results are shown in Tables 10–15.

In order to compare the effect of using self-encoding more intuitively, the following will average the results on different data sets, as shown in Figures 15–19.

Observing Tables 10–15, we can find that, in the five hyperparameter optimization methods, using self-encoding network to process data can improve the accuracy of the model, which reflects the superiority of data dimensionality reduction. Moreover, when comparing the hyperparameter optimization methods using self-encoding, the various indicators of the model under the WPA-PSO method are still the best, indicating that the hybrid algorithm has more powerful search and optimization capabilities than a single algorithm.

## 5. Conclusions

Based on the deep neural network for defect prediction, the article proposes a hybrid Wolf Pack algorithm to optimize the hyperparameters of the model, which enhances the model's global optimization and software defect prediction capabilities and performs data dimensionality reduction based on autoencoding to improve training and defect prediction effect. In order to prevent overfitting, this paper uses the early stopping method to stop the model when the training results are stagnant, such as when the continuous training brings little improvement or the continuous rounds of training do not bring any improvement. This can avoid only improving the index of the training set but lowering the index of the test set.

In future research, we can consider using other learning algorithms in deep learning to extract features and build software defect prediction models and compare the effectiveness of different learning algorithms.

## Figures and Tables

**Figure 1:** Basic rocket ship design. The rocket ship is propelled with three thrusters and features a single viewing window. The nose cone is detachable upon impact.

**Figure 2:** C language software measurement and defect data generation process.

**Figure 3:** Deep neural network structure.

**Figure 4:** Deep neural network structure.

**Figure 5:** Example of an autoencoder.

**Figure 6:** The flow chart of optimizing hyperparameters by hybrid Wolf Pack algorithm.

**Figure 7:** Flow chart of building software defect prediction model.

**Figure 8:** Flow chart of feature extraction based on AE.

**Figure 9:** CW4 experimental results histogram.

**Figure 10:** LR1 experimental results histogram.

**Figure 11:** PC5 experimental results histogram.

**Figure 12:** PC6 experimental results histogram.

**Figure 13:** PU1 experimental results histogram.

**Figure 14:** SF1 experimental results histogram.

**Figure 15:** Self-coding optimization comparison of grid searches.

**Figure 16:** Self-coding optimization comparison of random searches.

**Figure 17:** Self-coding optimization comparison of PSO.

**Figure 18:** Self-coding optimization comparison of WPA.

**Figure 19:** Self-coding optimization comparison of WPA-PSO.

**Table 1:** Commonly used software metrics for process-oriented software.

Category	Metrics
McCabe metrics	Cyclomatic complexity (*v*(*g*))
	Essential complexity (ev(*g*))
	Module design complexity (iv(*g*))
Halstead metrics	Unique operators (*n*_1_)
	Unique operands (*n*_2_)
	Total operators (*N*_1_)
	Total operands ( *N*_2_)
	Vocabulary (*n*)
	Length (*N*)
	Program volume (*V*)
	Program difficulty (*D*)
	Program level (Lv)
	Intelligence (*I*)
	Programming effort (*E*)
	Programming time (*T*)
LOC metrics	LOCphy
	LOComment
	LOBlank
	LOCComment
Reformatted code information for file	Total source lines
	Expansion factor
Procedure information	Average length of basic blocks
	Procedure entry points
	Procedure exit points
Comments associated with procedures	Total comments
	Comments in headers
	Comments in declarations
Ratio of comments to executable lines	Executable reformatted lines
	Total comments/Executable lines
	Header comments/executable lines
	Declaration comments/executable lines
	Code comments/executable lines
Complexity metrics	Knots
Loop/interval analysis	Number of loops
	Depth of loop nesting
	Number of order 1 intervals
	Maximum interval nesting
	Reducible intervals
LCSAJ and unreachability	Total LCSAJs
	Reachable LCSAJs
	Unreachable LCSAJs
	Maximum LCSAJ density
	Unreachable lines
	Unreachable branches
Dataflow information	Globals in procedure
	File fan in
	Fan out

**Table 2:** Temperature and wildlife count in the three areas covered by the study.

	Predictive value	
Defective module	Correct positive example (TP)	False positive (FP)
No defective modules	False negative (FN)	Correct negative example (TN)

**Table 3:** C project data set.

Data set	Number of samples	Number of defects	Defect rate (%)
CW4	1343	249	18.54
LR1	1078	133	12.34
PC5	423	39	9.22
PC6	846	63	7.45
PU1	1700	111	6.5
SF1	2731	353	12.93

**Table 4:** CW4 experimental results.

	Precision	Recall rate	F-measure	AUC
Grid	0.44	0.17	0.23	0.58
Random	0.54	0.21	0.29	0.60
PSO	0.61	0.27	0.37	0.62
WPA	0.65	0.33	0.43	0.64
WPA_PSO	0.73	0.36	0.48	0.67

**Table 5:** LR1 experimental results.

	Precision	Recall rate	F-measure	AUC
Grid	0.51	0.32	0.36	0.64
Random	0.50	0.30	0.31	0.63
PSO	0.57	0.46	0.50	0.71
WPA	0.61	0.53	0.56	0.74
WPA-PSO	0.62	0.58	0.59	0.77

**Table 6:** PC5 experimental results.

	Precision	Recall rate	F-measure	AUC
Grid	0.21	0.06	0.09	0.53
Random	0.18	0.08	0.10	0.53
PSO	0.37	0.31	0.33	0.63
WPA	0.45	0.43	0.43	0.69
WPA-PSO	0.52	0.49	0.48	0.72

**Table 7:** PC6 experimental results.

	Precision	Recall rate	F-measure	AUC
Grid	0.13	0.09	0.11	0.54
Random	0.51	0.38	0.42	0.68
PSO	0.71	0.49	0.57	0.73
WPA	0.72	0.53	0.61	0.75
WPA-PSO	0.73	0.55	0.62	0.76

**Table 8:** PU1 experimental results.

	Precision	Recall rate	F-measure	AUC
Grid	0.56	0.15	0.21	0.57
Random	0.75	0.24	0.34	0.62
PSO	0.81	0.44	0.56	0.71
WPA	0.85	0.50	0.62	0.75
WPA-PSO	0.86	0.55	0.67	0.77

**Table 9:** SF1 experimental results.

	Precision	Recall rate	F-measure	AUC
Grid	0.69	0.26	0.38	0.62
Random	0.71	0.28	0.40	0.63
PSO	0.67	0.36	0.45	0.66
WPA	0.72	0.42	0.52	0.69
WPA-PSO	0.73	0.49	0.59	0.73

**Table 10:** CW4 experimental results.

	Precision	Recall rate	F-measure	AUC
Grid	0.44	0.17	0.23	0.58
Grid + self-encoding	0.62	0.23	0.33	0.60
Random	0.54	0.21	0.29	0.60
Random + self-encoding	0.64	0.27	0.35	0.62
PSO	0.61	0.27	0.37	0.62
PSO + self-encoding	0.67	0.33	0.44	0.65
WPA	0.65	0.33	0.43	0.64
WPA + self-encoding	0.67	0.34	0.44	0.65
WPA_PSO	0.73	0.36	0.48	0.67
WPA_PSO + self-encoding	0.73	0.38	0.50	0.68

**Table 11:** LR1 experimental results.

	Precision	Recall rate	F-measure	AUC
Grid	0.51	0.32	0.36	0.64
Grid + self-encoding	0.61	0.39	0.47	0.68
Random	0.50	0.30	0.31	0.63
Random + self-encoding	0.60	0.35	0.43	0.66
PSO	0.57	0.46	0.50	0.71
PSO + self-encoding	0.64	0.56	0.59	0.76
WPA	0.61	0.53	0.56	0.74
WPA + self-encoding	0.64	0.57	0.60	0.76
WPA_PSO	0.62	0.58	0.59	0.77
WPA_PSO + self-encoding	0.62	0.64	0.62	0.79

**Table 12:** PC5 experimental results.

	Precision	Recall rate	F-measure	AUC
Grid	0.21	0.06	0.09	0.53
Grid + self-encoding	0.53	0.18	0.25	0.58
Random	0.18	0.08	0.10	0.53
Random + self-encoding	0.54	0.20	0.28	0.59
PSO	0.37	0.31	0.33	0.63
PSO + self-encoding	0.54	0.40	0.44	0.68
WPA	0.45	0.43	0.43	0.69
WPA + self-encoding	0.58	0.48	0.51	0.72
WPA_PSO	0.52	0.49	0.48	0.72
WPA_PSO + self-encoding	0.57	0.54	0.54	0.75

**Table 13:** PC6 experimental results.

	Precision	Recall rate	F-measure	AUC
Grid	0.13	0.09	0.11	0.54
Grid + self-encoding	0.42	0.27	0.33	0.63
Random	0.51	0.38	0.42	0.68
Random + self-encoding	0.70	0.45	0.53	0.71
PSO	0.71	0.49	0.57	0.73
PSO + self-encoding	0.72	0.53	0.61	0.75
WPA	0.72	0.53	0.61	0.75
WPA + self-encoding	0.73	0.56	0.63	0.77
WPA_PSO	0.73	0.55	0.62	0.76
WPA_PSO + self-encoding	0.74	0.56	0.64	0.77

**Table 14:** PU1 experimental results.

	Precision	Recall rate	F-measure	AUC
Grid	0.56	0.15	0.21	0.57
Grid + self-encoding	0.83	0.24	0.34	0.62
Random	0.75	0.24	0.34	0.62
Random + self-encoding	0.87	0.43	0.56	0.71
PSO	0.81	0.44	0.56	0.71
PSO + self-encoding	0.86	0.49	0.61	0.74
WPA	0.85	0.50	0.62	0.75
WPA + self-encoding	0.91	0.53	0.67	0.76
WPA_PSO	0.86	0.55	0.67	0.77
WPA_PSO + self-encoding	0.87	0.58	0.69	0.79

**Table 15:** SF1 experimental results.

	Precision	Recall rate	F-measure	AUC
Grid	0.69	0.26	0.38	0.62
Grid + self-encoding	0.71	0.29	0.40	0.64
Random	0.71	0.28	0.40	0.63
Random + self-encoding	0.71	0.34	0.46	0.66
PSO	0.67	0.36	0.45	0.66
PSO + self-encoding	0.70	0.41	0.51	0.69
WPA	0.72	0.42	0.52	0.69
WPA + self-encoding	0.75	0.48	0.58	0.73
WPA_PSO	0.73	0.49	0.59	0.73
WPA_PSO + self-encoding	0.76	0.52	0.62	0.75

## Data Availability

The data used to support the findings of this study are available at https://github.com/justlz/hybird-PSO-WPA/branches.
